The article "Influence of data mining technology in information analysis of human resource management on macroscopic economic management" was retracted in 2023. Reasons: unreliable results or conclusions; concerns about the peer review.

# Influence of data mining technology in information analysis of human resource management on macroscopic economic management

**DOI:** 10.1371/journal.pone.0251483

**Published:** 2021-05-18

**Authors:** Ai Zhang

**Affiliations:** Gannan University of Science and Technology, Ganzhou, China; Ministry of Natural Resources North Sea Bureau, CHINA

## Abstract

The purposes are to manage human resource data better and explore the association between Human Resource Management (HRM), data mining, and economic management. An Ensemble Classifier-Decision Tree (EC-DT) algorithm is proposed based on the single decision tree algorithm to analyze HRM data. The involved single decision tree algorithms include C4.5, Random Tree, J48, and SimpleCart. Then, an HRM system is established based on the designed algorithm, and the evaluation management and talent recommendation modules are tested. Finally, the designed algorithm is compared and tested. Experimental results suggest that C4.5 provides the highest classification accuracy among the single decision tree algorithms, reaching 76.69%; in contrast, the designed EC-DT algorithm can provide a classification accuracy of 79.97%. The proposed EC-DT algorithm is compared with the Content-based Recommendation Method (CRM) and the Collaborative Filtering Recommendation Method (CFRM), revealing that its Data Mining Recommendation Method (DMRM) can provide the highest accuracy and recall, reaching 35.2% and 41.6%, respectively. Therefore, the data mining-based HRM system can promote and guide enterprises to develop according to quantitative evaluation results. The above results can provide a reference for studying HRM systems based on data mining technology.

## Introduction

With the continuous reform and development of the economic system, enterprises’ development and competition are also changing continually. Moreover, the competition model has also shifted from material resource-based to human resource-based. Thus, Human Resource Management (HRM) has become a critical link for enterprises [1,2]. The HRM system takes human resource planning as the basis. It can provide an overall judgment on the enterprises’ internal employees’ information through the unified collection and management of employee information [3,4]. Manual HRM is not only time-consuming and labor-intensive but also prone to significant errors. Therefore, computer information technology has been introduced to solve this problem. Data mining technology has developed rapidly in recent years. It is a data analysis method characterized by the ability to extract potential information and knowledge. The statistical analysis methods, induction methods, spatial clustering methods, spatial analysis methods, rough set theory, and fuzzy set theory are well-known data mining algorithms [5,6]. Due to its excellent performance in processing massive data, the data mining technology has an extensive application scope. The decision tree algorithm is one of the essential methods among the classification analysis based on data mining. It can obtain the corresponding classification rules based on each tree branch [7,8].

Regarding the application of data mining technology in management systems, Marozzo et al. (2018) applied cloud software technology to describe the design and implementation of the data mining cloud framework. They found that the system can integrate visual workflow language with software service models to minimize the programming workload [9]. Zaborski et al. (2019) applied data mining algorithms, including artificial neural networks and classification regression trees, to analyze and research the prediction of reproduction parameters [10]. Shakil et al. (2020) investigated the developmental process of HRM and supply chain management informatization. They analyzed relevant research on the Scopus database using scientific analysis tools, classified and discussed the results, and further explored HRM informatization [11]. Sunmin et al. (2018) combined geographic information system tools and data mining models to analyze the relationship between flood-hit areas and related hydrological elements. By establishing data description factors in a spatial database, they found that the application of data mining could help further analyze economic and social activities and population and building density. Also, data mining could play a positive role in improving economic sustainability [12]. The above research shows the data mining has been applied to system management in many fields, and research results have been obtained. Its impact on the economy has been revealed; however, big data application in HRM analysis is rarely reported.

Hence, the ensemble classifier that integrates four decision tree algorithms is proposed to construct the HRM system, in an effort to find an approach suitable for data mining in HRM analysis. Then, the application potential of data mining in HRM and economic management can be revealed through the performance analysis of the algorithm and the characterization of the assessment management and the talent recommendation modules in the HRM system. The innovative point is the weighted integration of multiple decision tree algorithms to make full use of different single decision tree algorithms’ advantages and improve the classifier’s effects.

## Methods

### Data mining technology and decision tree algorithm

Data mining refers to the process of extracting potentially useful information from large quantities of random data. It is different from traditional data analysis methods. This method can mine and analyze information based on unclear assumptions, and the extracted information is effective, practical, and previous-unknown [13,14]. This technology is regarded as an information processing method from a business perspective. The analysis of business data has a close connection with the regulation and development of the macroscopic economy. Data mining technology can play a regulating role in the macroscopic economy. Data mining technology’s purpose is association analysis, classification prediction, and cluster analysis from a functional point of view. Specifically, correlation analysis aims to find the correlation network from the database. Classification can describe and predict the rules, in which decision trees are one of the principal methods. Cluster analysis is based on similarity, summarizing relevant data into different categories before analyzing them [15,16]. Because of the various types of data involved in HRM, decision tree algorithms’ application and effectiveness are discussed herein.

Data mining achieves classification by creating and using the classifiers. The decision tree algorithms utilize the mapping relationship between objects’ attributes and values, describe and analyze such mapping relationships using decision trees. The classification rules in the decision tree are formed by the interconnection between the root node and the leaf node, where the leaf node corresponds to the classification result. The ID3 algorithm is developed based on the decision tree learning idea. It is based on information gain and has been widely accepted since it was proposed. However, it also has some limitations in the application process. Therefore, the optimized C4.5 algorithm is proposed. Unlike the ID3 algorithm, the optimized algorithm is based on the information gain rate, which is also the uttermost difference between the ID3 and C4.5 algorithms in attribute selection metrics [17–19]. From the perspective of information theory and classification problems, the entropy *H(C)* can be expressed as:

$$H\left(C\right)=\sum_{i=1}^{n}p\left(c_{i}\right)\log_{2}p_{i}$$ (1)

In (1), *C* represents the category set, *c*_*i*_ denotes the value derived from the category set, *p* expresses the probability of appearance or occurrence of the category, and *n* signifies the number of categories. The information gain of the ID3 algorithm characterizes the degree of entropy fluctuation. Assuming that there is attribute *a*, and the elements contained in *B* are divided into *M* different subsets. At this time, the divided information entropy *H*_*a*_*(B)* can be described as:

$$H_{a}\left(B\right)=\sum_{j=1}^{m}\frac{\left|B_{j}\right|}{\left|B\right|}\times H\left(B_{j}\right)$$ (2)

Then the equation of information gain *IG(a)* can be obtained:

$$IG\left(a\right)=H\left(B\right)-H_{a}\left(B\right)$$ (3)

The optimal classification basis can be obtained based on the information gain with different attributes. The information gain rate can be obtained by calculating the split information *SI*_*a*_:

$$SI_{a}\left(B\right)=-\sum_{j=1}^{m}\frac{\left|B_{j}\right|}{\left|B\right|}\times \log_{2}\left(\frac{\left|B_{j}\right|}{\left|B\right|}\right)$$ (4)

Therefore, the equation corresponding to the information gain rate is expressed as:

$$IGA\left(a\right)=\frac{IG\left(a\right)}{SI\left(a\right)}$$ (5)

Since the C4.5 algorithm is based on the information gain rate, the offset problem caused by the information gain can be solved, the continuous attributes can be discretized, and the incomplete data can be processed. These are all the advantages of the C4.5 algorithm over the ID3 algorithm. Hence, the C4.5 algorithm is used as the fundamental algorithm in the HRM system information analysis.

### Data mining ensemble classifier based on Weka platform

As enterprises’ organizational structure develops, many enterprises have established human resource databases. Hence, the past manual analytical approaches cannot meet the needs of enterprise development. HRM data contain loads of vital economic knowledge and enterprise development patterns. Therefore, it is necessary to analyze HRM data using data mining techniques to find the hidden relationships and laws. Clustering analysis is a fundamental data mining approach that can automatically classify concrete or abstract objects as per the similarity; hence, the objects within the class have the highest similarity. Therefore, applying this approach to HRM can provide objective decision-making support for enterprise talent selection, employment, training, and other practical works. Among the learning software based on data mining, Weka has relatively complete data processing tools. It has applicability in different data mining algorithms. Specifically, its processing tools include data preprocessing, classification, association rules, and clustering [20,21]. In short, Weka is a data mining platform with multiple functions. It can also develop data mining functions based on its open-source interface. This tool can enable users to have a deeper understanding of data mining functions.

The ensemble classifier is composed of multiple base classifiers. Research results have revealed the ensemble classifier’s superior performance at the classification accuracy level compared to a single base classifier. Specifically, a group of differentiated base classifiers can be formed based on the determined training dataset, and the class label corresponding to the test dataset is predicted, thereby obtaining a sequence of corresponding classification results. The Bagging idea [22] is regarded as the foundation for constructing the ensemble classifier to improve the classification accuracy of single decision tree algorithm C4.5. In addition to the C4.5 algorithm, three decision tree algorithms: Random Tree [23], J48 [24], and SimpleCart, are also introduced to construct the ensemble classifier. The ensemble classifier’s implementation based on the above four decision tree algorithms is displayed in Fig 1 below.

**Fig 1:** Implementation of ensemble classifier based on four decision tree algorithms.

Data from the HRM system, mostly about enterprise, talent, and human resources, undergo data cleaning, data integration, and data conversion successively in the ensemble classifier model. According to the Bagging method, the training data set is randomly sampled with replacement to form four different training sets, written as *T*_*1*_, *T*_*2*_, *T*_*3*_, and *T*_*4*_. The weight value is 0.3 to make it convenient to explore the common weight of all classifiers. Next, four different decision tree classifiers are generated by Random Tree, J48, SimpleCart, and C4.5 algorithms successively, recorded as *C*_*1*_, *C*_*2*_, *C*_*3*_, and *C*_*4*_. The classification results can be obtained via each base classifier, and finally, the prediction function sequence can be formed. On this basis, each classification accuracy predicted by each base classifier is weighted, and the obtained classification results are voted. The weighting processing is described as:

$$C\left(w\right)=\underset{c\in \left\{1,2,3,\cdots ,C\right\}}{\arg\;\max}\sum_{i=1}^{M}\beta_{i}\cdot 1_{\left\{C_{i}\left(w\right)=c\right\}}$$ (6)

In (6), *C(w)* represents the classification weight, *C*_*i*_ represents the base classifier, and *β*_*i*_ represents the prediction accuracy. The larger the accuracy of the corresponding base classifier, the greater the value of the weight, The C4.5 parameters set are summarized in Table 1.

**Table 1:** Parameter setting of the C4.5 algorithm.

Parameter	Value
Criterion	entropy
Splitter	best
Pruning strategy	Min_samples_leaf
Post-pruning algorithm	REP
Target weight parameter	Min_weight_fraction_leaf

### Data mining-based HRM system

In the HRM field, the model based on manual data input and analysis is no longer applicable with the continuous expansion of data coverage, showing a series of drawbacks and limitations. Although the traditional data analysis methods can provide high data reliability and human analysis results, problems such as low efficiency, long research duration, and difficulty in data acquisition cannot be ignored. Moreover, due to the massive workload in the process, the traditional manual analysis methods can affect the relevant region’s economic development. Based on the above description of data mining technology and the design of ensemble classifier, data mining methods are introduced into the HRM system. The critical architecture of the system includes the collection system, database system, and management system. Data are stored and called via the interaction of various modules. The system composition of the proposed ensemble classifier based on data mining in the HRM system is shown in Fig 2 below.

**Fig 2:** System composition of ensemble classifier based on data mining in HRM system.

The assessment management module of the HRM system is the focus of analysis and evaluation. This module includes five submodules: department management, personnel management, recruitment management, performance assessment, and promotion management. The data mining technology is applied in the performance assessment submodule. In this module, especially the recruitment management sub-module, the recommendation of talents is also an important aspect. All human resources websites can provide the service of talent recommendation. The two methods that are commonly used for talent recommendation are CRM and CFRM, respectively. CRM has developed maturely; its overall implementation includes project feature extraction, feature model learning, and recommendation generation. Its users are independent and less affected by each other.

Most importantly, the cold start problem does not exist. However, CRM has problems such as the difficulty of extracting ideal features, the difficulty of mining users’ potential interests, and the cold start of the users, making it have greater limitations in applications. Compared with CRM, CFRM pays more attention to user participation and contribution. In the meantime, this method implements recommendations based on user interests. Its overall implementation includes scoring matrix creation, similarity calculation, and recommendation generation. CFRM can describe complex things while also being able to discover users’ potential preferences.

Nevertheless, it still has problems in matrix sparseness, cold start, and system scalability. Thus, the recommendation results of CRM and CFRM are not very effective. Hence, the data mining technology is introduced to the talent recommendation function in the HRM system due to its superiority in data processing.

The data mining-based talent recommendation method proposed above is recorded as DMRM. The data mining-based Ensemble Classifier-Decision Tree (EC-DT) algorithm is introduced into DMRM. The rigid filtering condition makes job recruitment more targeted and can effectively filter job applicants who do not meet the requirements. In addition, in the recommendation module, the job applicant’s characteristics are compared with non-rigid conditions, and the similarity is calculated. The specific equation is:

$$sim\left(N,C\right)=\cos\left(\vec{N},\vec{C}\right)=\frac{\vec{N}\cdot \vec{C}}{\left\|\vec{N}\right\|\left\|\vec{C}\right\|}$$ (7)

In (7), *N* represents a non-rigid condition, and *C* represents a condition that the job applicant has. Next, the weight of job application intention is calculated, and the corresponding equation is:

$$W_{i}=\sum_{p=1}^{n}v_{pq},q\in \left\{1,2,\cdots ,m\right\}$$ (8)

In (8), *W*_*i*_ refers to the position weight corresponding to the pre-recommended position under the number *i*, and *v*_*pq*_ represents the proportion of the position attribute *p* corresponding to the *q*-th value. After further standardization, the equation for the weight of job application intention can be expressed as:

$$NW_{i}=\frac{W_{i}-W_{\min}}{W_{\max}-W_{\min}}$$ (9)

In (9), *NW* represents the standardized weight, *W*_*min*_ describes the lower limit of the weight in the pre-recommended position, and *W*_*max*_ refers to the weight’s upper limit. Then the final weight can be calculated using the following equation:

$$FW_{i}=cw_{1}\cdot sim_{i}+cw_{2}\cdot N\left(W_{i}\right)$$ (10)

In (10), *FW*_*i*_ corresponds to the final weight of the position to be recommended under number *i*, *sim*_*i*_ refers to the non-rigid condition similarity of the position corresponding to *i*, *N(W*_*i*_*)* represents the standardized job application intention weight of the position corresponding to i, *cw*_*1*_ signifies the control weight parameter corresponding to the similarity, and *cw*_*2*_ stands for the control weight parameter corresponding to the intention weight.

### System test and analysis

Here, the classification accuracy serves as an indicator to verify the effectiveness of the data mining algorithm. The single Random Tree, J48, SimpleCart, and C4.5 algorithms are compared and analyzed with the EC-DT algorithm. The number of selected training samples is 5,000, and the number of test samples is 500. The experimental environment is Win 10, and the platforms are WEKA and UtraEdit. Data are collected from the HRM statistical data of ten listed enterprises.

CRM and CFRM are included for comparative analysis to verify the effectiveness of the proposed DMRM based on data mining. The selected evaluation indicators are precision and recall, respectively. The equation of CRM is:

$$\mathrm{Pr}ecision=\frac{CRN}{RN}$$ (11)

In (11), *CRN* represents the correct number of recommended positions, and *RN* represents the number of all positions in the recommended list. CFRM can be expressed as:

Recall=CRNTSN (12)

In (12), *CRN* represents the correct number of recommended positions, and *TSN* represents the number of all positions in the test set.

The EC-DT algorithm is selected to analyze the assessment management module in the HRM system. The selected indicators include team spirit (TS), sense of responsibility (R), creation spirit (CS), working ability (WA), morality and deeds (MD), communication and coordination (CC), and cost awareness (CA) [25]. The classification effect is evaluated by scoring results.

## Results and discussion

### Algorithm classification performance

The comparison results of four single decision tree algorithms and EC-DT algorithm based on the evaluation indicator of classification accuracy are presented in Fig 3 below.

**Fig 3:** Comparison results of single decision tree algorithms and EC-DT.

As shown in Fig 3, the changing trends of several classification algorithms under different samples are consistent. The classification accuracy of the EC-DT algorithm based on the ensemble classifier is significantly better than other decision tree algorithms. Among the single decision tree algorithms, the C4.5 algorithm can provide a higher classification accuracy than other algorithms. Specifically, the average classification accuracy rates of Random Tree, J48, SimpleCart, and C4.5 algorithms are 73.31%, 74.21%, 74.71%, and 76.69%, respectively. In contrast, the average classification accuracy of the ensemble classifier-based EC-DT algorithm is 79.97%. As the number of samples increases, the classification accuracy of the classifier first decreases and then increases. Fundamentally, when the number of samples is less than 1,500, the samples cannot display the data information features they have; moreover, as the number of samples increases, the classifier needs to record more sample information features a decrease in classification accuracy quickly. When the number of samples is greater than 1,500, the classifier can analyze and record the sample data’s information characteristics to increase the classifier’s accuracy. When the number of samples exceeds 3,800, some classifiers’ accuracy decreases again because the increase in samples leads to classifier overfitting, affecting the classifier’s accuracy.

Thus, it is reasonable to choose the C4.5 algorithm as the core classification algorithm. Moreover, the ensemble classifier plays a positive role in promoting the decision tree classification, and the obtained classification prediction results are the best. This result also shows that in addition to improving prediction accuracy, the algorithm’s generalization performance and robust performance can also be enhanced by combining weaker classifiers of different categories to form a better performance classifier.

### Personalized recommendation results based on data mining

The talent recommendation results obtained by CRM, CFRM, and DMRM are compared in precision and recall. The results are shown in Fig 4(A) and 4(B) below.

**Fig 4:** Comparison of talent recommendation results: (a) precision; (b) recall.

As shown in Fig 4, DMRM based on the proposed EC-DT algorithm has the highest recommendation precision. Specifically, when the recommendation list has 50 positions, CRM can provide a precision of 28.2%, CFRM can provide a precision of 26.3%, while DMRM can provide a precision of 35.2%. In terms of recall, DMRM based on the proposed EC-DT algorithm also presents the best performance. Specifically, when there are 50 positions in the recommendation list, the recall for CRM is 31.8%, the recall for CFRM is 30.9%, and the recall for DMRM can reach 41.6%. In comparison, personalized recommendation results based on ensemble classifier are the best, followed by CRM. The least effective recommendation method is CFRM.

Because CFRM is greatly affected by the sparse matrix, coupled with the particularity of the composition information of the job search, the lack of job evaluation leads to the reduction of recommendation accuracy, and the overall recommendation effect is not satisfactory. As for the CRM, due to the comparatively diversified composition of job information, the difficulty of extracting features increases, so that the recommendation effect of the algorithm becomes worse. In addition, the excessive dependence on the user background also leads to the effect deterioration of CRM. As the recommendation list positions increase, the recall also appears to be reduced, closely connected to the difficulty in digging the users’ potential and valuable information. In contrast, the proposed EC-DT personalized recommendation algorithm gives full play to data mining technology characteristics so that user information selection becomes more scientific and practical. In the meantime, it can also mine the potential information of users effectively. This is the reason that this algorithm can significantly improve precision and recall.

### Information analysis of HRM system

The HRM data of ten listed enterprises are selected for experiments. These enterprises are named as letters A to J. Seven indicators are chosen to assess data mining application in HRM, namely, Team Spirit (TS), Responsibility (R), Creativity Spirit (CS), Work Ability (WA), Morally Disengage (MD), Communication and Coordination (CC), and Cost Awareness (CA). The statistical results of the scores obtained according to the HRM system are presented in Fig 5 below.

**Fig 5:** Scoring statistics of the HRM assessment management module. (a) TS and R indicator scores. (b) CS and WA indicator scores. (c) MD, CC, and CA indicator scores.

The statistical results show that the HRM assessment module can provide a clear perception of the organizations’ overall situation. The quantitative scoring results reveal the actual level of each component or element in the enterprises or organizations, which can contribute to the development of the organizations. For example, Organization C has a TS score of 4, an R score of 2, and a CS score of 4, which are lower among the seven key evaluation indicators. Hence, Organization C can optimize and improve itself in this direction in subsequent development. In the meantime, this statistical result also reveals the importance of data mining methods in the information analysis of complex systems.

Enterprises’ development and macroscopic economic development complement each other. The development of enterprises even affects the development of the entire country’s economy. HRM is undoubtedly a key component in enterprise development. The development of enterprises depends on talents, and the introduction of talents depends on the continuous improvement and progress of the HRM system. The appropriate technological methods are of great significance to economic development under the rapid development of modern information techniques. Here, the decision tree algorithm in the data mining method is essentially applied. The effectiveness of the data mining method based on the ensemble classifier in HRM is verified through comparative analysis, which also illustrates the positive effect of data mining technology on macroscopic economic management.

## Conclusions

To analyze the HRM data using data mining techniques, an integrated classifier decision tree algorithm is designed by integrating four single decision tree algorithms, which dramatically improves the decision trees’ information processing ability. Then, the designed algorithm is applied to the evaluation management and talent recommendation of HRM. Test results reveal that the designed algorithm can improve data information classification accuracy, reaching 79.97%, a significant improvement compared with the single decision tree algorithm. The designed EC-DT algorithm can provide a recommendation accuracy rate of 35.2%, which can accurately recommend job applicants, proving the effectiveness of data mining techniques applied to HRM. Still, there are some weaknesses. The designed EC-DT can optimize the classification effect by adjusting the weight. Hence, studying the weight changes’ influences on the classification effect can further improve the algorithm’s cumulative effect. In the future, neural networks can optimize the integrated classifier to improve its effectiveness in processing HRM data.

## Supporting information

S1 Data (RAR)
